The article "Study on Risk Factors Related to Intrauterine Adhesion Based on Meta-Analysis" was retracted in 2023. Reasons: signs of a paper mill; compromised peer review; unreliable results or conclusions.

# Study on Risk Factors Related to Intrauterine Adhesion Based on Meta-Analysis

**DOI:** 10.1155/2022/4667679

**Published:** 2022-10-11

**Authors:** Sijing Li

**Affiliations:** Department of Hysteroscopic Centre, Fu Xing Hospital, Capital Medical University, Beijing 100038, China

## Abstract

**Objective:**

Intrauterine adhesion (IUA) is a severe complication that occurs following abortion. To evaluate the related risk factors of uterine cavity adhesion by meta-analysis.

**Methods:**

The research literature on the influencing factors of patients with intrauterine adhesions published from January 2010 to December 2020 in PubMed, EMBASE, Cochrane Library, web of science, CNKI, Wanfang Data, VIP, and CBM were retrieved by computer. Two evaluators independently screened the literature, extracted the data, and evaluated the treatment according to the inclusion and exclusion criteria and then analyzed it with revman5.3 software.

**Results:**

Finally, 12 literatures were included, with a total sample size of 2341 cases. The results of meta-analysis showed that pelvic inflammation (*p* = 0.05), negative pressure during uterine suction (*p* < 0.0001), and uterine suction time (*p* < 0.00001) were the risk factors for uterine cavity adhesion. The combined or and 95% CI of each factor were 2.05 (1.24, 3.38), 125.61 (67.35, 183.87), and 4.52 (4.21, 4.84), respectively. However, the number of pregnancies, the number of curettages, the average number of births, abortion, myomectomy, menstrual abnormalities, and infertility have little impact on the occurrence of intrauterine adhesions (*p* > 0.05).

**Conclusion:**

Pelvic inflammatory disease, negative pressure during uterine suction and uterine suction time are the risk factors leading to uterine cavity adhesion.

## 1. Introduction

Intrauterine adhesion (IUA), also known as Asherman's syndrome, is a common uterine disease that puzzles women of childbearing age. IUA is a disease that cannot repair itself after the endometrial basal layer is damaged, resulting in partial or complete closure of the uterine cavity and/or cervical canal [1], which is common in various invasive surgical procedures and infections in the uterine cavity. The main pathological change of IUA is that the normal endometrial tissue is replaced by the new fibrous scar tissue after the endometrial basal layer is damaged [2]. IUA is mainly manifested by menstruation reduction or amenorrhea, periodic lower abdominal pain related to menstrual cycle, abortion, infertility, etc. With the increase of invasive uterine procedures such as induced abortion and the full liberalization of the national policy of two and three births, the prevalence of IUA also showed an obvious upward trend. The report shows that the incidence of intrauterine adhesion after abortion is 19.1%, which is positively correlated with the number of intrauterine operations such as curettage [3]. IUA seriously affects the physical, mental, and reproductive health of women, makes patients face a heavy psychological and economic burden, and brings many family and social problems. Its diagnosis and treatment has been widely concerned [4, 5]. The causes of IUA include dilatation/curettage, postpartum hemorrhage, myomectomy, hysteroscopic surgery, and genital tuberculosis. At present, the treatment for IUA is hysteroscopic adhesiolysis [6], but there is still a high recurrence rate after this treatment method [7]. Previous clinical studies on the related risk factors of patients with intrauterine adhesions are mostly retrospective studies, and there is no relevant meta-analysis report.

Therefore, this study aimed to collect relevant literature at home and abroad and to evaluate the related factors affecting postoperative pregnancy of patients with intrauterine adhesions through meta-analysis.

## 2. Materials and Methods

### 2.1. Literature Search

By searching the research literature on the influencing factors of postoperative pregnancy in patients with intrauterine adhesions published in PubMed (PubMed, https://pubmed.ncbi.nlm.nih.gov), Excerpta Medica Database (EMBASE, https://www.embase.com), Cochrane Library, Web of Science (https://www.cochranelibrary.com), Chinese National Knowledge Infrastructure (CNKI, https://en.cnki.com.cn), Wanfang Data (https://www.wanfangdata.com.cn), the Chongqing VIP Chinese Science (VIP, http://cqvip.com), and China Biomedical Literature Database (CBM, https://www.sciencedirect.com/topics/nursing-and-health-professions/chinese-biomedical-database) from January 2010 to December 2020. Chinese key words: “intrauterine adhesion,” “risk factors,” “influencing factors,” “related factors,” etc. English search terms: “Asherman syndrom,” “influencing factor,” “risk factor,” “related factor,” etc. Endnote X9 was applied to document management and weight removal, and the documents that may meet the inclusion criteria were determined by manual filtration.

### 2.2. Literature Screening and Data Extraction

Inclusion criteria are as follows: (1) domestic and foreign published case-control studies or retrospective studies or current situation studies on the relevant risk factors of patients with intrauterine adhesions, which are divided into case groups and control groups and compared according to their exposure factors; (2) intrauterine adhesions confirmed by hysteroscopy; and (3) if it is a document published by the same author in different years, select the one with better quality.

Exclusion criteria are as follows: (1) repeated published literature, systematic evaluation, review, meta-analysis, case report; and (2) the data in the study are incomplete or inaccurate.

### 2.3. Document Extraction and Quality Evaluation

Two researchers independently extracted the title, author, publication date, and outcome indicators for verification. If two researchers disagree, it will be decided by the third party. The Newcastle Ottawa scale (NOS) recommended by Cochrane Collaboration Network was used to evaluate the quality of literature, including the selection of research objects, comparability between groups, and outcomes [8]. 7-9 were high-quality literature, 5-6 were medium quality literature, and 0-4 points are low-quality literature.

### 2.4. Statistical Methods

RevMan 5.3 software was used to analyze all the data of this study [9], and *p* < 0.05 was considered to be statistically significant. *Q* test and *I*^2^ were used to test the heterogeneity of the included literature. If *I*^2^ < 50% or *p* > 0.05, it was considered that there was no heterogeneity between the studies, and the fixed effect model was used for analysis; otherwise, the random effect model is used. Funnel plot is used to analyze the publication bias. If the funnel plot is asymmetrically distributed, Begg rank correlation method is used to further test the publication bias of this study [10]. If *p* < 0.05, it is considered that there is a potential publication bias. If *p* > 0.05, it is considered that there is no publication bias.

## 3. Results

### 3.1. Basic Information of Literature

After searching the relevant database, a total of 1876 literatures were obtained, and all of them were imported into endnote software. According to the established literature inclusion and exclusion criteria and literature quality control requirements, a total of 12 literatures were finally included in this study [11–22], all of which were retrospective analysis, with a total of 2341 patients. The document screening process was shown in Figure 1. The basic characteristics of the study were shown in Table 1.

### 3.2. Effect of Pelvic Inflammation on Intrauterine Adhesion

A total of 2 studies were included [16, 21]. The heterogeneity test showed that *I*^2^ = 72%, *p* = 0.06, had no obvious heterogeneity found, and the fixed effect model was used. The results of meta-analysis were shown in Figure 2. Pelvic inflammatory disease was a risk factor for uterine cavity adhesion (OR = 2.05, 95% CI: 1.24~3.38), which was statistically significant (*p* = 0.005).

### 3.3. Effect of Pregnancy Times on Intrauterine Adhesion

A total of 7 studies were included [14–16, 19–22]. The heterogeneity test showed that *I*^2^ = 97%, *p* < 0.00001, with obvious heterogeneity. The random effect model was used. The results of meta-analysis were shown in Figure 3. The number of pregnancies had little effect on the occurrence of intrauterine adhesion (OR = 0.47, 95% CI: -0.35~1.29), which was not statistically significant (*p* = 0.26).

### 3.4. Effect of Negative Pressure on Intrauterine Adhesion during Uterine Suction

A total of two studies were included [21, 22]. The heterogeneity test showed that *I*^2^ = 97%, *p* < 0.00001, with obvious heterogeneity, using the random effect model. The results of meta-analysis were shown in Figure 4. Negative pressure during uterine aspiration was a risk factor for patients with intrauterine adhesion (OR = 125.61, 95% CI: 67.35~183.87), which was statistically significant (*p* < 0.0001).

### 3.5. Effect of Uterine Suction Time on Intrauterine Adhesion

A total of three studies were included [18, 21, 22]. The heterogeneity test showed that *I*^2^ = 99%, *p* < 0.00001, with obvious heterogeneity, using the random effect model. The results of meta-analysis were shown in Figure 5. The time of uterine aspiration was a risk factor for patients with intrauterine adhesion (OR = 4.52, 95% CI: 4.21~4.84), which was statistically significant (*p* < 0.00001).

### 3.6. Effect of Curettage Times on Intrauterine Adhesion

A total of 3 studies were included [15, 20, 21]. The heterogeneity test showed that *I*^2^ = 97%, *p* < 0.00001, with obvious heterogeneity, using the random effect model. The results of meta-analysis were shown in Figure 6. The number of curettages had little effect on the occurrence of intrauterine adhesion in patients (OR = 0.48, 95% CI: -0.63~1.60), and was not statistically significant (*p* = 0.40).

### 3.7. The Effect of Average Birth Times on Intrauterine Adhesion

A total of 3 studies were included [14, 19, 21]. The heterogeneity test showed that *I*^2^ = 98%, *p* < 0.00001, with obvious heterogeneity, and the random effect model was used. The results of meta-analysis were shown in Figure 7. The average number of births had little effect on the occurrence of intrauterine adhesions (OR = 0.44, 95% CI:-0.14~1.02) and was not statistically significant (*p* = 0.14).

### 3.8. Effect of Abortion on Intrauterine Adhesion

A total of 6 studies were included [11, 12, 16, 17, 19, 20]. The heterogeneity test showed that *I*^2^ = 63%, *p* = 0.02, with obvious heterogeneity. The random effect model was used. The results of meta-analysis were shown in Figure 8. Abortion had little effect on the occurrence of intrauterine adhesion (OR = 1.08, 95% CI: 0.63~1.85) and was not statistically significant (*p* = 0.77).

### 3.9. Effect of Myomectomy on Intrauterine Adhesion

The heterogeneity test of two studies [12, 19] showed that *I*^2^ = 19%, *p* = 0.27, no obvious heterogeneity was found, and the fixed effect model was used. The results of meta-analysis are shown in Figure 9. Myomectomy had little effect on the occurrence of intrauterine adhesion (OR = 1.35, 95% CI: 0.39~4.67) and was not statistically significant (*p* = 0.63).

### 3.10. Effect of Abnormal Menstruation on Intrauterine Adhesion

A total of 3 studies were included [13, 15, 20]. The heterogeneity test showed that *I*^2^ = 92%, *p* < 0.00001, with obvious heterogeneity, and the random effect model was used. The results of meta-analysis were shown in Figure 10. Abnormal menstruation had little effect on the occurrence of intrauterine adhesions (OR = 0.83, 95% CI: 0.09~7.36) and was not statistically significant (*p* = 0.87).

### 3.11. Effect of Infertility on Intrauterine Adhesion

The heterogeneity test that included two studies [13, 19] showed that *I*^2^ = 81%, *p* = 0.02, with obvious heterogeneity, using random effect model. The results of meta-analysis were shown in Figure 11. Infertility had little effect on the occurrence of intrauterine adhesion (OR = 0.51, 95% CI: 0.06~4.00) and was not statistically significant (*p* = 0.52).

### 3.12. Publication Bias Analysis

As shown in Figure 12, the funnel plot analysis of publication bias showed that the funnel plot was symmetrically distributed, indicating that there was no significant publication bias in the included studies.

## 4. Discussion

Intrauterine adhesion is mainly caused by the damage of the endometrium caused by surgery, which will not only affect the menstrual cycle, but also lead to fibrinogen exudation and other phenomena. In clinical practice, patients are often accompanied by irregular menstruation, abdominal pain, and other phenomena. If measures are not taken in time, amenorrhea and infertility may also occur. Therefore, it will have a greater impact on those with fertility needs [23]. The female uterine wall is relatively soft, so the operator must strictly grasp the depth when carrying out the curettage operation. If multiple curettage interventions are required, it will not only prolong the time of uterine suction but also increase the negative pressure during uterine suction, which will increase the probability of damaging the endometrial basal layer. Therefore, it is easy to have intrauterine adhesion after abortion [24]. It can be seen that there are many risk factors leading to intrauterine adhesions. The results of meta-analysis of this study showed that pelvic inflammation (OR = 2.05, 95% CI: 1.24~3.38, *p* = 0.005), negative pressure during uterine suction (OR = 125.61, 95% CI: 67.35~183.87, *p* < 0.0001) and uterine suction time (OR = 4.52, 95% CI: 4.21~4.84, *p* < 0.00001) were the risk factors leading to intrauterine adhesions, which were supported by previous studies [25–27]. However, the number of pregnancies (OR = 0.47, 95% CI: -0.35~1.29, *p* = 0.26), the number of curettages (OR = 0.48, 95% CI: -0.63~1.60, *p* = 0.40), the average number of births (OR = 0.44, 95% CI:-0.14~1.02, *p* = 0.14), abortion (OR = 1.08, 95% CI: 0.63~1.85, *p* = 0.77), myomectomy (OR = 1.35, 95% CI: 0.39~4.67, *p* = 0.63), menstrual abnormalities (OR = 0.83, 95% CI: 0.09~7.36, *p* = 0.87), and infertility (OR = 0.51, 95% CI: 0.06~4.00, *p* = 0.52) had little impact on the occurrence of intrauterine adhesions.

The degree of intrauterine adhesion is serious, the clinical treatment effect is poor, and the postoperative pregnancy rate is low. The possible reason is that endometrial damage and tissue fibrosis are serious, endometrial regeneration mechanism is destroyed, and neovascularization is blocked, resulting in endometrial stromal cells and epithelial cells regeneration obstacles, and it is difficult to achieve self-repair [28]. From the perspective of clinical research, many gynecological diseases and operations easily lead to intrauterine adhesion, which has a great impact on women's health. From the perspective of pathogenesis, it is because the female endometrial basal layer is injured, such as surgical trauma or inflammation, which affects the normal menstrual cycle. Endometrial abscission causes interstitial fibrinogen leakage at the same time, and after deposition at the gap, it leads to adhesion between the anterior and posterior walls of the uterine cavity [29]. Generally, women with intrauterine adhesions will suffer from abdominal pain, abnormal menstruation, and abnormal pregnancy. With the development of the disease, if not controlled in time, it will also lead to amenorrhea, oligomenorrhea, and periodic abdominal pain. In serious cases, it will lead to infertility and bring great damage to women, especially infertile women [30]. With the improvement of medical technology in China, more and more experts began to choose hysteroscopy to assist in the treatment of intrauterine adhesions. Through hysteroscopy, we can clearly observe the specific situation of intrauterine adhesion of patients, and then select the appropriate surgical instruments for operation. This advanced surgical method has the characteristics of simple operation, less trauma, less bleeding, and fast postoperative healing [31]. However, before hysteroscopic surgery, it is necessary to grade the degree of intrauterine adhesion of patients and make corresponding preparations to improve the surgical effect [32].

The database included in this study only contained 8 Chinese and English databases, and the search results were lacking on foreign related research, which may lead to incomplete literature included in the study and affect the stability of meta-analysis results. In addition, the included studies were of small sample size, single center clinical control studies, which lacked the support of multi center, and large sample size studies, which may increase the occurrence of bias.

## 5. Conclusion

To sum up, pelvic inflammation, negative pressure during uterine suction, and uterine suction time are the risk factors for uterine cavity adhesion. This meta-analysis suggests that there are many risk factors for intrauterine adhesion. The more serious the pelvic inflammation, the greater the negative pressure during uterine suction, and the longer the time of uterine suction, the higher the risk of intrauterine adhesion. The results of this study provide new insights into the prevention of IUA.

## Figures and Tables

**Figure 1:** Document screening flow chart.

**Figure 2:** Effect of pelvic inflammation on intrauterine adhesion.

**Figure 3:** Effect of pregnancy times on intrauterine adhesion.

**Figure 4:** Effect of negative pressure on intrauterine adhesion during uterine suction.

**Figure 5:** Effect of uterine suction time on intrauterine adhesion.

**Figure 6:** Effect of curettage times on intrauterine adhesion.

**Figure 7:** Effect of average number of births on intrauterine adhesion.

**Figure 8:** Effect of abortion on intrauterine adhesion.

**Figure 9:** Effect of myomectomy on intrauterine adhesion.

**Figure 10:** Effect of abnormal menstruation on intrauterine adhesion.

**Figure 11:** Effect of infertility on intrauterine adhesion.

**Figure 12:** Funnel diagram.

**Table 1:** Basic characteristics of included literature.

Author	Years	*N*		Risk factors	NOS scores
		Experience group	Control group		
Ajayi et al. [11]	2017	265	641	(7)	6
Dawood et al. [12]	2010	30	24	(7) (8)	8
Liu et al. [13]	2014	50	10	(9) (10)	9
Can et al. [14]	2018	31	29	(2) (6)	7
Zhu et al. [15]	2019	180	56	(2) (5) (9)	5
Li et al. [16]	2019	48	52	(1) (2) (7)	6
Mentula et al. [17]	2018	12	80	(7)	8
Ludwin et al. [18]	2014	47	49	(4)	8
Chen et al. [19]	2015	29	53	(2) (6) (7) (8) (10)	7
Zhu et al. [20]	2018	74	76	(2) (5) (7) (9)	5
Du and Wang [21]	2020	66	339	(1) (2) (3) (4) (5)	9
He [22]	2020	50	50	(2) (3) (4) (6)	8

Note: (1) pelvic inflammation; (2) pregnancy times; (3) negative pressure during uterine suction; (4) suction time; (5) number of curettages; (6) average number of births; (7) abortion; (8) myomectomy of uterus; (9) abnormal menstruation; (10) infertility.

## Data Availability

Data generated in this study are available from the corresponding author under reasonable requests.
